The article "Predictors of frequent oral analgesic use in rheumatoid arthritis" was published in 2014. Journal: Pak J Med Sci.

# Predictors of frequent oral analgesic use in rheumatoid arthritis

**DOI:** 10.12669/pjms.305.5112

**Published:** 2014

**Authors:** Esha das Gupta, Huey Shin Tee, Rajalingham Sakthiswary

**Affiliations:** 1 Esha das Gupta, Department of Medicine, International Medical University, Jalan Rasah, 70300 Seremban, Negeri Sembilan, Malaysia.; 2 Huey Shin Tee, Department of Medicine, International Medical University, Jalan Rasah, 70300 Seremban, Negeri Sembilan, Malaysia.; 3 Rajalingham Sakthiswary, Department of Medicine, Universiti Kebangsaan Malaysia Medical Centre, 56000 Cheras, Malaysia.

**Keywords:** Analgesic, Rheumatoid arthritis

## Abstract

***Objective: ***The main objective of this study was to determine the predictors of frequent oral analgesic use among Rheumatoid Arthritis (RA) patients who were prescribed with the above medication on an ‘as-needed’ basis.

***Methods: ***Patients with RA were recruited consecutively from the Rheumatology outpatient clinics in this cross-sectional study. The sociodemographic data, frequency of oral analgesic intake, Patient Global Assessment (PGA) scores and HAQ (Health Assessment Questionnaire) scores were determined by interviewing the subjects. Subjects were divided into 2 groups; frequent users (3 days and above in a week) and less frequent users (less than 3 days in a week).

***Results: ***In a total of 112 subjects, 39 (34.8%) were frequent analgesic users. Both the HAQ and PGA scores were significantly higher among the frequent users (p<0.05). Using multivariate analysis, the HAQ scores (p=0.015, odds ratio 3.161 [95% confidence interval of 1.246-8.015]) and PGA scores (p=0.039 odds ratio 1.291 [95% confidence interval of 1.012-1.646]) were found to be independent predictors of frequent analgesic use.

***Conclusions:*** Our study confirms that the frequency of analgesic intake in Rheumatoid Arthritis has a significant relationship with patient-reported functional capacity and well being.

## INTRODUCTION

Rheumatoid Arthritis is a chronic inflammatory disease which causes polyarticular pain compromising the well-being and quality of life of the sufferers.^1^^,^^2^ Although there has been a surge in the number of disease modifying anti rheumatic drugs (DMARDS) in the recent years, oral analgesics continue to be an intergral part of RA treatment.^3^ The frequency of analgesic intake is a subjective measure of disease activity in clinical practice. 

The oral analgesics which are widely prescribed in RA are paracetamol and non-steroidal anti inflammatory drugs (NSAIDs).^4^^,^^5^ In patients with mild to moderate disease activity, analgesics are often prescribed on an ‘as-needed” basis.

Apart from imposing additional costs in the treatment of RA, oral analgesics especially NSAIDs are associated with several side effects such as analgesic nephropathy, gastric ulcer and cardiovascular events.^6^^-^^8^ In 1983, the estimated direct medical costs of arthritis treatment in the USA was $8.6 billion and a further $3.9 billion was spent on treating gastrointestinal side-effects of NSAIDs, giving rise to a total of $12.5 billion.^4^

Apart from the intensity of pain, there are other factors which could potentially influence the frequency of analgesic use.^5^^,^^9^ Female gender, for instance, was associated with increased use of analgesics in a study involving community-dwelling older people with chronic non-malignant pain.^10^ Poor self-rated fitness, age and smoking were related to a continuous regular analgesics use in a population-based Danish study.^11^ The subject on pattern and use of analgesics in RA has not received the attention it deserves from a research perspective. Research on painkillers in RA has traditionally placed much emphasis and focused on adherence to analgesics^12^ including methods of measuring compliance.^13^ The main objective of this study, was therefore, to determine the predictors of frequent analgesic use in RA.

## METHODS

***Study Design and population: ***This was a cross-sectional, monocentric study conducted at the Tuanku Jaafar Hospital in Seremban, Malaysia between September and December 2012. Subjects were recruited consecutively from the Rheumatology outpatient clinics. The following were the inclusion criteria of this study;

1. Patients diagnosed with Rheumatoid Arthritis based on American College of Rheumatology 1987^14^ or 2010.^15^
2. Patients aged 18 years and above.
3. Patients who have taken analgesics for joint pain anytime during the one month period prior to the study.
4. Patients who were prescribed with oral analgesics on an “as-needed’ basis
5. Patients who were able to read, write and understand English.

The following patients were excluded: 1. Patients who had functional disability due to neurological disorders such as stroke, muscular dystrophy, Parkinson’s disease and spinal cord compression. 2. Patients who took analgesics for pain at sites apart from the joints such as abdominal pain, headache and pelvic pain. Written consent was taken from all patients who fulfilled the above mentioned criteria and agreed to participate in this study. 

The frequency of oral analgesic intake for the purpose of this study was based on the average number of days in a week the subject had consumed the drug in the one month period prior to the study. Based on this parameter, subjects were divided into 2 groups; frequent users (3 days and above in a week) and less frequent users (less than 3 days in a week). 

***Data Collection: ***The medical records of all subjects were reviewed to gather information on the disease duration and list of medications; particularly DMARDs (both conventional and biologic agents) and oral analgesics. The socio demographic data, frequency of oral analgesic intake, Patient Global Assessment (PGA) scores and Stanford HAQ (Health Assessment Questionnaire) 8-Item Disability Scale scores were determined by interviewing the subjects. In the field of rheumatology, one of the most popular and widely used self-reported measures of physical disability is the Stanford Health Assessment Questionnaire Disability Index (HAQ-DI).^16^ The Stanford HAQ 8-Item Disability Scale consists of 8 questions regarding the limitations patients experience in performing their daily activities. Patients were asked how difficult it was to perform an activity on a scale of 0 (without any difficulty) to 3 (unable to do). The scores based on the 8 questions were averaged to construct a single total score.

The Patient Global Assessment (PGA) required patients to rate how they felt overall using a scale of 0 (very well) to 10 (very poor). Previous studies have proven that PGA has good (0.702) test-retest reliability in RA.^17^

***Statistical Analysis: ***Data were analysed using the Statistical Package for Social Sciences (SPSS) package for Windows version 21. Continuous variables were expressed as mean ± SD. Categorical variables were analysed using the chi square exact test whereas the Mann-Whitney test and Independent T test were used for continuous variables. The odds ratio (OR) was determined using binary logistic regression for variables with significant p values (p<0.05) on univariate analysis. Linear regression analysis was performed to determine the relationship between a continuous dependent variable and a continuous explanatory variable.

## RESULTS

***Sociodemographic and Clinical Data: ***In a total of 112 subjects, 39 (34.8%) were frequent analgesic users based on our study definition of 3 days and above in a week. The demographic and clinical characteristics of the frequent users and less frequent users are summarised in Table-I. The vast majority of the patients included in this study were females (81.3%). The mean age of the subjects was 53.6 years. There were no significant differences between the two groups in demographic, disease duration, use of DMARDs, use of complimentary medicine and number of joints with synovitis. NSAIDs and Paracetamol were the most frequently used analgesics among the frequent users (74.3%) and the less frequent users (50.7%), respectively. A significantly higher percentage of less frequent analgesic users (67.1%, p=0.049) were able to perform basic activities of daily living (ADL) independently. Early Morning Stiffness which is a subjective marker of inflammatory activity in RA^18^ was more common among the frequent users although statistical significance in the difference was not reached. 

***Patient-reported Measures: ***The patient-reported measures i.e Stanford HAQ 8-Item Disability Scale and PGA are described in Table-II. Both the HAQ and PGA scores were significantly higher among the frequent users (p<0.05). The above mentioned variables were further analysed using logistic regression model. The HAQ scores (p=0.015, odds ratio 3.161 [95% confidence interval of 1.246-8.015]) and PGA scores (p=0.039 odds ratio 1.291 [95% confidence interval of 1.012-1.646]) were independent predictors of frequent analgesic use. The HAQ scores (p<0.05, standardized beta coefficient 0.514), but not the PGA scores (p=0.055, standardized beta coefficient 0.172) had a significant positive correlation with the number of days in a week of analgesic use (Fig.1). 

## DISCUSSION

In this study, we have explored the factors influencing frequent oral analgesic intake among RA patients who were prescribed with the above therapy on an ‘as-needed’ basis. The novel findings of this study are that the 2 patient-reported measures (PGA and HAQ scores) are independent predictors of frequent oral analgesic use in RA. Functional capacity as reflected by the HAQ scores had a significant association and positive correlation with the frequency of analgesic use.

**Table-I:** Comparison of sociodemographic, clinical and functional characteristics between frequent and less frequent analgesic users

***Variable***	***Frequent Users*** ***(n=39)***	***Less frequent Users*** ***(n=73)***	***p value***
Age (years), Mean ± SD	54.05 ± 13.18	53.56 ± 10.88	0.834
*Gender, n(%)*			
Male	9 (23.1)	12 (16.4)	0.231
Female	30 (76.9)	61 (83.6)	
*Race, n(%)*			
Malay	9 (23.1)	21 (28.8)	0.805
Chinese	10 (25.6)	18 (24.7)	
Indian	19 (48.7)	32 (43.8)	
Others	1 (2.6)	2 (2.7)	
Average income (Ringgit Malaysia) Median (range)	850 (4860)	1000(8000)	0.188
*Occupation, n(%)*			
Unemployed/Housewife	15 (38.5)	30 (41.1)	0.419
Professional	12 (30.8)	23 (31.5)	
Non professional	1 (2.6)	11 (15.1)	
Retired	3 (7.7)	9 (12.3)	
*Disease Duration, n (%)*			
<1 year	6 (15.4)	4 (13.7)	0.227
1-5 years	17(43.6)	25 (34.2)	
6-10 years	6 (15.4)	21 (28.8)	
10-20 years	6 (15.4)	15 (20.5)	
>20 years	4 (10.2)	8 (11.0)	
Conventional DMARDS only, n(%)	31 (79.5)	60 (75.9)	0.398
Biologics, n(%)	4 (10.3)	8 (10.9)	0.347
Complimentary Medicine, n(%)	12 (30.8)	16 (21.9)	0.199
*Most Frequently Taken Analgesic, n(%)*			
Paracetamol	10 (25.6)	37 (50.7)	0.084
NSAIDs	29 (74.3)	34 (46.6)	
Tramadol	0 (0)	2 (2.7)	
Independent in basic ADLs, n(%)	16 (41.0)	49 (67.1)	0.049
Early morning stiffness of >half an hour, n (%)	17 (43.6)	24 (32.9)	0.180
*No. of joints with physician observed synovitis, n (%)*			
0	2 (5.1)	6 (8.2)	0.578
1-2	7 (17.9)	20 (27.4)	
3-5	13 (33.3)	16 (21.9)	
>5	17 (43.6)	31 (42.5)	

DMARDS: disease modifying antirheumatic drugs, ADL: activities of daily living.

**Table-II:** Comparison of Patient-Reported Measures between the Study Groups

**Variable**	**Frequent Users** **(n=39)**	**Less frequent Users** **(n=73)**	**p value**
*HAQ score Mean ± SD	0.87 ± 0.58	0.39 ± 0.48	<0.05
*Dress yourself, n(%)*			
0	17 (43.6)	48 (65.8)	0.026
1	16 (41.6)	17 (23.3)	
2	4 (10.3)	4 (5.5)	
3	2 (5.1)	3 (4.1)	
*Get in and out of bed, n(%)*			
0	21 (53.8)	47 (64.4)	0.282
1	12 (30.8)	18 (24.7)	
2	6 (15.4)	7 (9.6)	
3	0 (0)	1 (1.4)	
*Lift a full cup or glass to your mouth, n(%)*			
0	26 (66.7)	56 (76.7)	0.722
1	8 (20.5)	9 (12.3)	
2	5 (12.8)	8 (11.0)	
3	0 (0)	0 (0)	
*Walk outdoors on flat ground, n(%)*			
0	23 (59.0)	47 (64.4)	0.282
1	13 (33.3)	17 (23.3)	
2	1 (2.6)	7 (9.6)	
3	2 (5.1)	2 (2.7)	
*Wash and dry your entire body, n(%)*			
0	25 (64.1)	58 (79.5)	0.103
1	11 (28.2)	10 (13.7)	
2	3 (7.7)	4 (5.5)	
3	0 (0)	1 (1.4)	
*Bend down to pick up clothing from the floor, n(%)*			
0	12 (30.8)	36 (49.3)	0.090
1	13 (33.3)	20 (27.4)	
2	12 (30.8)	10 (13.7)	
3	2 (5.1)	7 (9.6)	
*Turn regular faucets on and off, n(%)*			
0	18 (46.2)	42 (57.5)	0.183
1	12 (30.8)	21 (28.8)	
2	8 (20.5)	9 (12.3)	
3	1 (2.6)	1 (1.4)	
*Get in and out of a car, bus, train or airplane, n(%)*			
0	14 (35.9)	41 (56.2)	0.019
1	15 (38.5)	25 (34.2)	
2	10 (25.6)	5 (6.8)	
3	0 (0)	2 (2.7)	
*Patient Global Assessment, Median (range)*	*6 (8)*	*5 (9)*	*<0.05*

**Fig.1:** Correlation between HAQ score and frequency of analgesic intake (number of days in a week).

There is a complex interplay of factors that influence pain severity and in turn, the patterns and frequency of analgesic use.^5^ Silva Luna et al.^19^ reported that higher HAQ scores were associated with worse scores of visual analogue scale for pain and higher scores on the subscale of negative mood. In fact, Sokka et al.^20^ concluded that HAQ scores correlated at higher levels with pain scores than with radiographic scores of small joints.

The HAQ score among the frequent-users were significantly higher despite a comparable number of joints with physician-observed synovitis in both the study groups (p=0.578). This finding suggests that functional capacity has a stronger link to pain perception, sensitivity and response compared to disease activity in RA. Along this line, many studies have highlighted that disease activity in RA may not necessarily correlate with measures of pain.^21^^,^^22^

PGA is one of the 4 components in the calculation of Disease Activity Score based on 28-joints (DAS28) for evaluation of disease activity in RA. Based on our findings, the PGA was an independent predictor of frequent analgesic use although it did not correlate significantly with the number of days in a week of analgesic use among the subjects. In keeping with our findings, Lati et al. concluded that PGA had the strongest association with pain and depressive symptoms in RA.^23^ Data from clinical trials have indicated that the PGA incorporates patient perceptions encompassing several aspects of pain management including the control of analgesic administration. Besides, PGA ratings were in the expected direction and parallel to other patient-reported outcome measures in various clinical studies involving other medical conditions.^24^

We do recognise and acknowledge the drawbacks of our study. The cross-sectional study design assumes that the frequency of analgesic use had remained stable for the one month period prior to the study. As the course of RA may fluctuate in some patients, the aforementioned parameter may not hold true over time. Mounting evidence assigns multifactorial influences with regard to pain sensitivity and response. We did not address other factors such as mood, psychometric properties of analgesic intake and the level of education. Moreover, the questionnaires were interviewer- assisted which may be more likely to result in biased response compared to self-completed questionnaires. However, a single interviewer was used throughout the study in an attempt to avoid inter-interviewer variability which may affect the study results. 

In conclusion, this study has identified 2 widely used patient-reported measures in RA clinical studies, namely HAQ and PGA scores as independent predictors of frequent analgesic use in RA. These findings which emphasize the importance of functional capacity and patients’ perception of well being in the use of analgesics; would hopefully be validated by larger, prospective studies in the near future. 

## Authors Contribution:

**EDG **conceived, designed and did statistical analysis & editing of manuscript.

**HST** and RS did data collection and manuscript writing.

## Notes

***Source of funding:*** None.

## References

[1] Odegard S, Finset A, Kvien TK, Mowinckel P, Uhlig T (2005). Work disability in rheumatoid arthritis is predicted by physical and psychological health status: a 7-year study from the Oslo RA register. Scand J Rheumatol.

[2] Smedstad LM, Moum T, Vaglum P, Kvien TK (1996). The impact of early rheumatoid arthritis on psychological distress. A comparison between 238 patients with RA and 116 matched controls. Scand J Rheumatol.

[3] Al MJ, Maniadakis N, Grijseels EW, Janssen M (2008). Costs and effects of various analgesic treatments for patients with rheumatoid arthritis and osteoarthritis in the Netherlands. Value Health.

[4] Bloom BS (1988). Cost of treating arthritis and NSAID-related gastrointestinal side-effects. Aliment Pharmacol Ther.

[5] Blamey R, Jolly K, Greenfield S, Jobanputra P (2009). Patterns of analgesic use, pain and self-efficacy: a cross-sectional study of patients attending a hospital rheumatology clinic. BMC Musculoskelet Disord.

[6] Giercksky KE, Huseby G, Rugstad HE (1989). Epidemiology of NSAID-related gastrointestinal side effects. Scand J Gastroenterol Suppl.

[7] Bluhm B, Green LA (2011). NSAID use associated with increased cardiovascular risk and death, but naproxen appears to be the least harmful. Evid Based Med.

[8] Ng SC, Chan FK (2010). NSAID-induced gastrointestinal and cardiovascular injury. Curr Opin Gastroenterol.

[9] Gustafsson M, Gaston-Johansson F, Aschenbrenner D, Merboth M (1999). Pain, coping and analgesic medication usage in rheumatoid arthritis patients. Patient Educ Couns.

[10] Kung F, Gibson SJ, Helme RD (1999). Factors associated with analgesic and psychotropic medications use by community-dwelling older people with chronic pain. Aust N Z J Public Health.

[11] Hargreave M, Andersen TV, Nielsen A, Munk C, Liaw KL, Kjaer SK (2010). Factors associated with a continuous regular analgesic use - a population-based study of more than 45,000 Danish women and men 18-45 years of age. Pharmacoepidemiol Drug Saf.

[12] Harrold LR, Andrade SE (2009). Medication adherence of patients with selected rheumatic conditions: a systematic review of the literature. Semin Arthritis Rheum.

[13] Rapoff MA, Belmont JM, Lindsley CB, Olson NY (2005). Electronically monitored adherence to medications by newly diagnosed patients with juvenile rheumatoid arthritis. Arthritis and rheumatism.

[14] Arnett FC, Edworthy SM, Bloch DA, McShane DJ, Fries JF, Cooper NS (1988). The American Rheumatism Association 1987 revised criteria for the classification of rheumatoid arthritis. Arthritis and rheumatism.

[15] Aletaha D, Neogi T, Silman AJ, Funovits J, Felson DT, Bingham CO, 3rd (2010). 2010 rheumatoid arthritis classification criteria: an American College of Rheumatology/European League Against Rheumatism collaborative initiative. Annals of the rheumatic diseases.

[16] Fries JF, Spitz P, Kraines RG, Holman HR (1980). Measurement of patient outcome in arthritis. Arthritis and rheumatism.

[17] Rohekar G, Pope J (2009). Test-retest reliability of patient global assessment and physician global assessment in rheumatoid arthritis. J Rheumatol.

[18] Yazici Y, Pincus T, Kautiainen H, Sokka T (2004). Morning stiffness in patients with early rheumatoid arthritis is associated more strongly with functional disability than with joint swelling and erythrocyte sedimentation rate. J Rheumatol.

[19] Silva Luna K, Ortiz AM, Patino E, Aguilera C, Velasco T, Garcia de Vicuna R (2012). Influence of the structure of mood in the assessment of rheumatoid arthritis through the visual analog scale for pain, HAQ and DAS28. Reumatol Clin.

[20] Sokka T, Kankainen A, Hannonen P (2000). Scores for functional disability in patients with rheumatoid arthritis are correlated at higher levels with pain scores than with radiographic scores. Arthritis Rheumatism.

[21] Celik S, Fresko I, Sut N, Batumlu NM, Yazici H, Yazici Y (2010). Differences in pain and fatigue perception among a group of rheumatoid arthritis patients in the United States and in Turkey who have similar disease activity and functional status. Clin Exp Rheumatol.

[22] Bostrom C, Harms-Ringdahl K, Nordemar R (1995). Relationships between measurements of impairment, disability, pain, and disease activity in rheumatoid arthritis patients with shoulder problems. Scand J Rheumatol.

[23] Lati C, Guthrie LC, Ward MM (2010). Comparison of the construct validity and sensitivity to change of the visual analog scale and a modified rating scale as measures of patient global assessment in rheumatoid arthritis. The Journal of Rheumatology.

[24] Rothman M, Vallow S, Damaraju CV, Hewitt DJ (2009). Using the patient global assessment of the method of pain control to assess new analgesic modalities in clinical trials. Curr Med Res Opin.

